The article "A Cohort Study to Assess Cognitive Impairment and Its Effects on Older Patients in the Orthopedic Rehabilitation" was published in 2022. Journal: J Healthc Eng.

# A Cohort Study to Assess Cognitive Impairment and Its Effects on Older Patients in the Orthopedic Rehabilitation

**DOI:** 10.1155/2022/7821525

**Published:** 2022-02-18

**Authors:** Han Zhang, Bo Pang, Zheng Ma, Huimei Dong, Hongyi He, Lan Jiang

**Affiliations:** Department of Rehabilitation Medicine, Shanghai Jiao Tong University Affiliated Sixth People's Hospital, Shanghai, China

## Abstract

**Background:**

The cognitive role of older patients is regularly not investigated in orthopedic rehabilitation, after the elective as well as the nonelective operation. The objective of this research is to investigate the cognitive disorder and its influence over the duration of stay along with the functional consequences of the older patients who were admitted to orthopedic rehabilitation. *Material and Methods*. The inclusion criteria for this study were the patients with age above 50 years; who were admitted with the detection of orthopedic impairment and the surgery both elective and nonelective, investigated utilizing the MoCA (Montreal Cognitive Assessment) over admission, MBI (Modified Barthel Index), and FIM (Function Independent Measure) over admission and discharge status; and were discharged from the hospital. The demography, as well as the clinical data, comprising of the duration of stay, age and the detection was also reported.

**Result:**

Of the 109 admitted patients, 80 patients were included in the study where *n* = 47 (58.75%) patients were females and *n* = 33 (41.25%) were males. The age group range was 50 to 94 years with a mean age of 78.5 years (SD = 8.27). The diagnostic groups included for the study were fractured neck of femur (*n* = 34; 42.5%), orthopedic surgery (*n* = 22; 27.5%), and other orthopedic surgery (*n* = 24; 30%). The mean duration of rehabilitation stay was reported as 34 (4.39), where the MoCA was reported as 22.17 (2.44); functional independence measures were as follows: motor admission as 53.97 (7.55), motor discharge as 76.27 (5.35), cognitive admission as 30.71 (1.99), and cognitive discharge as 31.85 (1.94). Here, the diagnosis was done over the fractured neck of the femur (i.e., NOF being 34 (42.5%), elective surgeries 22 (27.5%), and other orthopedic as 24 (30%)).

**Conclusion:**

An excessive percentage of older-age patients in a rehabilitation unit with elective as well as nonelective diagnoses comprises the cognitive disorder. The cognitive screening was advised for all the older age patients in the rehabilitation units to report a specific rehabilitation plan to enhance the consequences along with the duration of stay. There is further study required to explore different cognitive strategies to enhance the rehabilitation consequences among older-age orthopedic patients.

The article "A Cohort Study to Assess Cognitive Impairment and Its Effects on Older Patients in the Orthopedic Rehabilitation" was published in 2022. Journal: J Healthc Eng.

## 1. Introduction

Cognitive impairment is a well-defined risk element for the damaging falls in older ages [1, 2]. As a consequence, it will be anticipated that chronic cognitive diseases like dementia or Alzheimer's are widely prevailing among older patients depending on multiple factors comprising of characteristic diagnostic parameters and the severity of the clinical manifestations. Postoperative cognitive disorders are frequently observed among elderly patients (age >65 years). These comprise mainly of degraded perception, information investigation, memory, concentrating strength, attention and focus, and the patient's response and reaction [3, 4].

The cases of cognitive disorders have been documented as independent risk measures for delirium, and the total case of the new delirium was remarkably observed higher among the older patients suffering from dementia, as compared to the older patients suffering from no dementia [5, 6]. Furthermore, the prefracture cognitive impairments along with the postfracture suffering of delirium were found to be strongly associated with the higher rate of mortality as well as the risk for the establishment, and the delirium may be an untimely indicator for the postdischarge cognitive degeneration [7, 8]. However, this can generate an outcome in the long-run cognitive degeneration, postoperative cognitive degeneration peripheral to the delirium which does not happen in all the patients.

The cognitive variations in the rehabilitation might be preexisting, which even may be an element causing orthopedic injury in a person [9, 10]. The rehabilitation from a therapy aspect might not individually focus on the cognitive impairment, instead, via the design of the rehabilitation program, assimilate the cognitive role to enhance the participation in the rehabilitation program, as a result of which improving the functional consequences [11]. The evidence proposes that the cognitively impaired suffering older patients can be benefitted from the specialized rehabilitation programs, which is more rigorous, with the patients with average-to-acute cognitive impairment determined to exhibit functional enhancements in the rehabilitation programs [12, 13].

The cognitive status can be a crucial predicting factor of the rehabilitation consequences, along with being aware of the information related to the cognitive abilities of the patient and the dimensions of deficiency facilitating the staff with the retrain in the useful task rendition, comprising of day-to-day activities like walking. To enhance the functional consequences of all the older patients with orthopedic conditions, a better comprehension of the cognitive abilities of the patient and how it can affect their process of rehabilitation is needed [14–16]. Various rehabilitation units implement the cognitive screens to help the decision-making procedure about both appropriateness of a patient who has to be admitted to a rehabilitation unit and the timing as well as assistance needed for discharge, although the screening tools implemented are not steady [17].

The article "A Cohort Study to Assess Cognitive Impairment and Its Effects on Older Patients in the Orthopedic Rehabilitation" was published in 2022. Journal: J Healthc Eng.

The objective of this study is to assess, through a cohort study, the association between the cognitions, calculated with the use of MoCA, and other functional outcomes, calculated using the FIM as well as the MBI, of the older patients with orthopedic condition, who were admitted into the rehabilitation, with the detection of the fractured neck of the femur, elective as well as other related orthopedic operations, and the duration of patient's stay [18]. The occupational therapists furnish the intervention associated to enhance the function in the orthopedic rehabilitation program. The occupational therapy involvement furnished the location of the study conducted and was constant beyond the detection, with the rehabilitation involvement specifically focusing on the requirements of the individuals.

It was hypothesized that the relation between the cognitive impairment and the consequences in the orthopedic rehabilitation may occur for the patients who were admitted with fracture injury, who inclined to be older and weaker, as compared to the ones who were admitted for the elective process.

## 2. Material and Methods

The audit was verified by the Research and the Ethics Committee, where the patients were recognized via the procedure of admission to the common rehabilitation unit. This unit was facilitated with the staff having a specialized multidisciplinary team, comprising physiotherapy, dietetics, social work, speech pathology, occupational therapy, and medical and nursing.

The inclusion criteria for this study were as follows: (1) the patients with age above 50 years; (2) the patients who were admitted with the detection of orthopedic impairment and the surgery both elective and nonelective, investigated utilizing the MoCA over admission, MBI as well as FIM over admission, and discharge status; and (3) the patients who were discharged from the hospital. The data for this cohort study was gathered through chart data entry and the status of admission and discharge data which is regularly gathered by the occupational therapy group.

The demography as well as the clinical data comprising of the duration of stay and age and the detection was also reported. The diagnosis was classified into subgroups: elective orthopedic surgery of hip as well as knee replacement, fractured neck of femur, and other associated orthopedic injuries comprising the orthopedic injury of the upper as well as the lower limbs along with the fractured pelvis.

The article "A Cohort Study to Assess Cognitive Impairment and Its Effects on Older Patients in the Orthopedic Rehabilitation" was published in 2022. Journal: J Healthc Eng.

The cognition was investigated over the admission utilizing the MoCA and the patients were classified into the groups of severity level as per the scale, to compare the variation between the diagnosis categorized in the range of 26 to 30 in the normal range followed by the range of 18 to 25 as the mild cognitive impairment, the score of 10 to 17 as the moderate cognitive impairment, and the score of 9 or below than that was the less severity of cognitive impairment.

Quantitative values were described using their number, mean, standard deviation, and median; MoCA scores on admission and discharge were compared using ANOVA with repeated measures, with age and education as covariables. Qualitative values were described using their number, frequencies, and centiles and were compared using the Chi^2^ test or Fisher's exact test when necessary. To evaluate the change in MoCA score as a function of its baseline value, we split the study population into three subgroups with low (≤21), intermediate (≥22 and ≤25), and high (≥26) MoCA scores. All analyses were performed using SPSS software V22.0 (IBM SPSS Inc., Armonk, NY, USA).

## 3. Results

### 3.1. Patients' Characteristics

A total of 109 patients were admitted to the rehabilitation center from January to August 2019 where people with orthopedic injuries and surgeries were selected. Out of these, 29 patients were excluded who did not meet the criteria for inclusion (for not completing the MoCA). Of the 109 admitted patients, 80 patients were included in the study where *n* = 47 (58.75%) patients were females and *n* = 33 (41.25%) were males.

The age group range was 50 to 94 years with a mean age of 78.5 years (SD = 8.27). The diagnostic groups included for the study were fractured neck of femur (*n* = 34; 42.5%), orthopedic surgery (*n* = 22; 27.5%), and other orthopedic surgery (*n* = 24; 30%). The surgeries elected were planned prior to or scheduled. The patient's characteristics are presented in Table 1.

The clinical characteristics of the subgroups which are selected for diagnosis are shown in Tables 1 and 2. Collective MoCA score for the diagnosis was found to show mild impairment. A significant difference in FIM scores (both cognitive and motor), MBI scores at the time of admission or discharge, age, and diagnosis type was noted.

The post hoc analysis showed a significant difference in the scores of cognition where surgery patient scores were higher significantly in comparison to the patients with fractured neck of femur, though there was no other difference between fractured NOF or other orthopedic surgery patients. Statistical analysis has also shown that the FIM scores of cognition between fractured NOF and elective surgery patients were different (0.367). There was no significant change noted between patients with fractured NOF or other orthopedic cases or with elective surgery.

The article "A Cohort Study to Assess Cognitive Impairment and Its Effects on Older Patients in the Orthopedic Rehabilitation" was published in 2022. Journal: J Healthc Eng.

### 3.2. Significance between MoCA and FIM Scores and Their Functional Outcomes

The functional analysis was done on the basis of the FIM scores (motor) at the time of admission and discharge as well as the MBI scores at the time of admission and discharge were assessed. At the time of admission, a significant change in the FIM motor scores was noted on the basis of the diagnosis type. The post hoc analysis noted that patients with elective orthopedic surgery had a score significantly higher than the NOF cases of patients and with other orthopedic cases of patients.

No significant changes were noted in the FIM scores (motor) at the admission time for patients with fractured neck of femur and other patients with orthopedic cases. The post hoc analysis also revealed that the scores of elective orthopedic patients were higher significantly when compared with patients with fractured neck of the femur or other orthopedic surgery. In the discharge FIM scores (discharge), no difference was noted between orthopedic patients and fractured NOF.

The analysis revealed that the MBI scores were showing a significant difference between fractured NOF and elective orthopedic patients (*P*=0.001). The analysis has no significant difference when MoCA scores showed no significant differences with the MBI change or FIM motor score (Table 2).

The median of MoCA for NOF and orthopedic surgery was 22 and that of other orthopedic surgeries was found to be 22. The median for FIM motor admission for NOF was 50.5, orthopedic surgery was 65, and another orthopedic surgery was found to be 50. The median for FIM cognition for admission in case of admission for NOF was 30, orthopedic surgery was 32.5, and another orthopedic surgery was 30, whereas the median for FIM cognition discharge for NOF was 31, orthopedic surgery was 33, and other orthopedic procedures was 30.

The median for FIM motor admission for NOF was found to be 71.5, orthopedic surgery was 81.5, and another orthopedic surgery was 76.5 (Table 2). MoCA scores and FIM cognition scores were compared against the functional variables where the association between cognition and discharge was linked significantly with the length of stay in the hospital. A marked association was seen in MoCA scores with FIM admission (motor), MBI discharge, and FIM admission/discharge (cognition, motor).

The article "A Cohort Study to Assess Cognitive Impairment and Its Effects on Older Patients in the Orthopedic Rehabilitation" was published in 2022. Journal: J Healthc Eng.

## 4. Discussion

In this study, it can be observed that a higher number of geriatric orthopedic older-age patients in the rehabilitation, in spite of the reason behind their admission, that is, either selective or nonselective operation, have experienced cognitive impairment (*n* = 80), as calculated by the MoCA. In this cohort analysis, we have indicated a median point with faint cognitive impairment, with fewer scores on the MoCA. The NOF group accounts for a larger proportion of fracture types and is associated with cognitive dysfunction in elective and other types of orthopaedic surgery.

There was zero significant variation found between the categories for their total MoCA scores, although there was a significant variation observed between the FIM cognitive score over the admission or the discharge status of patients, thus indicating the lower functional cognition of the patients with a fractured NOF as well as the other orthopedic status. With the scope of diagnosis for other orthopedic states and fractured NOF category, it can be presumed that these were because of the drops for which the precognitive state might have furnished to the risk of fall down.

The MBI was outstandingly varied between the three diagnoses, signifying that the calculation of function via observation, comprising of FIM as well as MBI, inspects the variations in the diagnostic categories. The FIM motor variations for all categories were considered clinically remarkable, thus assisting its implementation as a functional result calculated, on an orthopedic rehabilitation department.

The MBI variation from the status of admission of a patient to the discharge was remarkably varied with the highest development prevailing in the other orthopedic category, densely followed by the fractured NOF category, assisting its utilization as a result measure of role among these patient populations. This also signifies that these patients experienced a better functional result, with alike cognitive capabilities to those allowed for the elective operation. As observed in other researches, the patients who were admitted with a fracture with a history of falls, usually had a failing function before their admission, which affects functional results, but it may even yield more chances for enhancement.

Furthermore, the patients who were admitted for elective operation might be prepared before admitting with social assistance, home set-up and on completion of the prior-admitting exercises, therefore possessing a greater initial point of function with slighter advancements quantifiable after the rehabilitation plan. Moreover, the results of MoCA, FIM movement variation, and MBI nonexpression did not help patients with severe cognitive impairment improvement during rehabilitation. However, a substantial specimen size with more practicality of cognition is needed.

The article "A Cohort Study to Assess Cognitive Impairment and Its Effects on Older Patients in the Orthopedic Rehabilitation" was published in 2022. Journal: J Healthc Eng.

The average duration of stay for those patients who were admitted with fracture NOF was a duration of 34 days and the other orthopedic patient for a duration of 36 days, while the elective orthopedic operation of the patients experienced a 34-day duration of stay. This was above and beyond the range of this project, although it might demonstrate the varied operations in rehabilitation or the patient parameters, like the high rate of cognitive impairment. This should be reported that the average age of these older patients who were admitted to these rehabilitation centers and assessed for this analysis was greater than the national average. Here, the national average age of orthopedic patients turns out to be 78.5 years (SD = 8.27).

The discoveries signify that all the cognitive computations, both MoCA and FIM cognitive scores, were linked with the duration of stay in the group total but not in individual diagnosis. This signifies that beyond both the elective and the nonelective orthopedic recognition, cognition can report the duration of stay. The correlation between cognition and hospitalization time shows that even the slightest reduction in cognition is also obvious, so it is necessary to reduce the cost of medical services.

This aids the advice of the cognitive partitions utilized with all the patients who are admitted to the geriatric orthopedic rehabilitation centers, despite the detection. This process of screening might help the programs to adapt how the rehabilitation is carried out, with respect to the functional context, specific prompts, as well as the assimilation of the cognitive training policies to make as large as possible for the functional results and then possibly diminish the duration of stay.

Cognition is majorly affected by age and it can impact the patient's potential to actively get involved in the process of rehabilitation goal setting, learning and deficient in the remembering skills, tough with the decision making the discharge site and the services needed. The outcomes signify that for the group of fractured NOF along with other groups of orthopedic, the MoCA scores were associated with the functional scores of the FIM (i.e., the admission and the discharge status) and the MBI (i.e., the discharge status), therefore signifying that the MoCA is functional in calculating the cognition before as well as after the rehabilitation as linked to the useful measures at both points.

The article "A Cohort Study to Assess Cognitive Impairment and Its Effects on Older Patients in the Orthopedic Rehabilitation" was published in 2022. Journal: J Healthc Eng.

Although, for the elective operation group, the FIM cognitive and not the MoCA, overadmitting was associated with the functional measures (i.e., FIM motor and the MBI over the admission of patients), but only the FIM motor overdischarge of patients. This proposes that for the elective operation group, the FIM cognitive is more functional in terms of measuring the cognitive potential, which will be associated with the functional behaviour.

There was no significant variation while drawing a comparison of the severity on the MoCA to the detection, and the breakdown of the scores on the basis of the assessing areas was further investigated, which would be advantageous to identify the aspects of cognition associated with the duration of stay. The MoCA scores and the location of discharge were found to be significantly different between those who were discharged directly to their homes and the ones discharged to any other location like a nursing center or an independent care unit or a hostel.

The details of specific cognitive deficiency were experienced by those patients who were admitted to the orthopedic units and would report the design of the rehabilitation program. Furthermore, with the fall as the primary reason for the orthopedic injury among the older patients, the fall prevention programs comprising of the education parameter were needed to count the cognitive elements to enhance their efficacy in lessening as well as preventing the falls. The experts promote the consideration of the role of technology in enhancing the results as well as the assistance of the older people to administer their process of rehabilitation.

Therefore, the implementation of the technology to report the rehabilitation for the people with cognitive modifications in orthopedic rehabilitation needs assessment. The additional study has to be conducted more efficiently to provide rehabilitation to those elder patients with orthopedic conditions, with cognitive impairment, who were likely excluded from the conducted rehabilitation trials.

## 5. Conclusion

To conclude, the geriatric patients with orthopedic conditions, who were admitted to the rehabilitation, were bestowed with the cognitive impairment beyond the detection and this was linked with the discharge location, useful outcomes, and the duration of stay. The cognitive screening is advised for all the older patients with orthopedic conditions who were admitted to the rehabilitation programs to report an individualized rehabilitation program in order to enhance the results and the duration of stay. Furthermore, the study is needed to investigate the cognitive plans to maximize the rehabilitation results among older patients with orthopedic conditions.

The article "A Cohort Study to Assess Cognitive Impairment and Its Effects on Older Patients in the Orthopedic Rehabilitation" was published in 2022. Journal: J Healthc Eng.

## Figures and Tables

**Table 1:** Clinical characteristics of patients included in the study.

S. no.	Characteristic	Mean
(1)	Rehabilitation length of stay	34 (4.39)

(2)	Male	33
	Female	47

(3)	Montreal cognitive assessment	22.17 (2.44)

(4)	*Functional independence measure*	
	Motor admission	53.97 (7.55)
	Motor discharge	76.27 (5.35)
	Cognitive admission	30.71 (1.99)
	Cognitive discharge	31.85 (1.94)

		Number (%)

(5)	*Diagnosis*	
	Fractured neck of femur (NOF)	34 (42.5)
	Elective surgeries	22 (27.5)
	Other orthopedic	24 (30)

**Table 2:** Detailed patient characteristics.

S. no.	Description	Fractured neck of femur (NOF) (*n* = 34)	Orthopedic surgery (*n* = 22)	Other orthopedic surgeries (*n* = 24)	*P* value
(1)	Age	50–9872.79 (8.48)	71–89 81 (4.93)	73–92 84.33 (4.47)	0.001^*∗*^

(2)	Length of stay	34 (4.48)	34 (3.38)	36 (4.90)	<0.001^*∗*^

(3)	*Montreal cognitive assessment (MoCA)*	*Median, IQR (n %)*			
	Median (IQR)	22 (17–25)	22 (17–25)	22 (19–25)	0.105
	Intact (*n*, %)	3 (8.82)	4 (18.18)	4 (16.66)	
	Mild (*n*, %)	14 (41.17)	13 (59.09)	11 (45.83)	
	Moderate (*n*, %)	9 (26.47)	3 (13.63)	8 (33.33)	
	Severe (*n*, %)	1 (2.94)	1 (4.45)	1 (4.16)	

(4)	*FIM motor*	*Median*	
	Admission	50.5 (43–58)	65 (56–70)	50 (42–55)	<0.001^*∗*^
	Discharge	71.5 (65–81)	81.5 (79–85)	76.5 (68–81)	<0.001^*∗*^
	Change	25 (14–30)	12–24 (20.5)	25 (10–30)	0.016

(5)	*FIM cognition*	*Median*	
	Admission	30 (26–33)	32.5 (29–34)	30 (27–34)	0.014^*∗*^
	Discharge	31 (28–35)	33 (30–35)	32 (29–34)	0.034^*∗*^
	Change	0–2	0–1	0–2	0.367^*∗*^

(6)	*MBI*				
	*Admission*				
	Minimal assistance	0	0	1 (4.16)	<0.001^*∗*^
	Mild dependence (*n* %)	12 (35.29)	7 (31.81)	12 (50)	
	Moderate dependence (*n* %)	15 (44.11)	11 (50)	7 (29.16)	
	Severe dependence (*n* %)	4 (11.76)	4 (18.18)	3 (12.5)	
	Total dependence (n %)	2 (5.88)	0	0	
	*Discharge*				
	Independent (*n* %)	2 (5.88)	6 (27.27)	3 (12.5)	0.001^*∗*^
	Minimal assistance (*n* %)	16 (47.05)	12 (54.54)	13 (5.42)	
	Mild dependence (*n* %)	9 (26.47)	2 (9.09)	4 (16.66)	
	Moderate dependence (*n* %)	5 (14.71)	1 (4.54)	3 (12.5)	
	Severe dependence (*n* %)	1 (2.94)	1 (4.54)	1 (4.16)	
	Total dependence (*n* %)	1 (2.94)	0	0	

## Data Availability

The data used to support this study are available from the corresponding author upon request.
